This article has been retracted.

# Transdermal delivery of allopurinol-loaded nanostructured lipid carrier in the treatment of gout

**DOI:** 10.1186/s40360-022-00625-y

**Published:** 2022-11-28

**Authors:** Zakir Ali, Fakhar ud Din, Fatima Zahid, Saba Sohail, Basalat Imran, Salman Khan, Maimoona Malik, Alam Zeb, Gul Majid Khan

**Affiliations:** 1 Nanomedicine Research Group, Department of Pharmacy, Quaid-I-Azam University, Islamabad, Pakistan; 2 Department of Pharmacy, Faculty of Biological Sciences, Quaid-I-Azam University, Islamabad, Pakistan; 3 Department of Pharmacy, Riphah International University, Islamabad, Pakistan; 4 Islamia College University, Peshawar, Pakistan

**Keywords:** Allopurinol, Nanostructured lipid carriers, Anti-gout study, Transdermal

## Abstract

**Background:**

Allopurinol (ALP), a xanthine oxidase inhibitor, is a first line drug for the treatment of gout and hyperuricemia. Being the member of BCS class II drugs, ALP has solubility problem, which affects its bioavailability. Also, ALP has shorter half-life and showed GI related problems. In present study, ALP was encapsulated in nanostructured lipid carriers (NLCs) to ensure enhanced bioavailability, improved efficacy and safety in vivo.

**Methodology:**

ALP-loaded NLCs were fabricated by micro-emulsion technique. The prepared NLCs were optimized via design expert in term of particle size, zeta potential and entrapment efficiency. FTIR, PXRD and TEM analysis were carried out to check chemical interaction, polymorphic form and surface morphology of the optimized formulation. ALP-loaded NLCs were then loaded into HPMC based poloxamer-407 gel and were characterized. In vitro and ex vivo analysis were carried out via dialysis membrane method and franz diffusion cell, respectively. Uric acid was used for induction of gout and the anti-gout activity of ALP-loaded NLCs gel was performed and compared with ALP suspension.

**Results:**

The optimized formulation had particles in nano-range (238.13 nm) with suitable zeta potential (-31.5 mV), poly-dispersity index (0.115) and entrapment of 87.24%. FTIR results confirmed absence of chemical interaction among formulation ingredients. XRD indicated amorphous nature of ALP-loaded NLCs, whereas TEM analysis confirmed spherical morphology of nanoparticles. The optimized formulation was successfully loaded in to gel and characterized accordingly. The in vitro release and drug release kinetics models showed sustained release of the drug from ALP-loaded NLCs gel. Furthermore, about 28 fold enhanced permeation was observed from ALP-loaded NLCs gel as compared to conventional gel. Skin irritation study disclosed safety of ALP-loaded NLCs gel for transdermal application. Furthermore, ALP-loaded NLCs gel showed significantly enhanced anti-gout activity in Sprague–Dawley rats after transdermal administration as compared to oral ALP suspension.

**Conclusion:**

ALP-loaded NLCs gel after transdermal administration sustained the drug release, avoid gastrointestinal side effects and enhance the anti-gout performance of ALP. It can be concluded, that NLCs have the potential to deliver drugs via transdermal route as indicated in case of allopurinol.

## Introduction

Gout is an inflammatory disease characterized by monosodium urate monohydrate (MSU) crystals deposition in synovial fluid and other tissues [1]. It is the most common inflammatory arthritis in men and a major cause of inflammatory arthritis in women after menopause [2]. In gout, both acute and chronic inflammatory responses are caused by nucleation, growth and apposition of monosodium urate crystals. Gout, when compared with other rheumatic diseases, has a unique feature that can reverse hyperuricemia which is the commonest pathophysiological mechanism for crystal formation. As the serum uric acid level is reduced below the solubility threshold, it result in the dissolution of MSU crystals leading to gout cure [3]. Allopurinol (ALP) is the structural isomer of hypoxanthine and was introduced in 1946 by Elion, et al. at the Burroughs–Wellcome Company [4]. It works by the inhibition of enzyme Xanthine oxidase, responsible for the formation of uric acid [5]. In 1966, it was approved by food and drug administration (FDA) for the treatment of gout and hyperuricemia and is the drug of choice and first line therapy in treatment of gout [6, 7]. It has been used in the treatment of gout and allied hyperuricemia condition (kidney stone and tumor lysis syndrome) for more than 50 years. Despite the 1^st^ line drug, ALP has the problem of insolubility in aqueous and acidic solutions. Also ALP has a shorter half-life of 1–2 h due to metabolism in liver. Both these factor limits the bioavailability of ALP, leading to its reduced choice as therapeutic agent [8, 9]. Also, ALP is associated with gastrointestinal side effect (vomiting, diarrhea), neurological signs (pain, drowsiness) and hypersensitivity (malaise, fever, eosinophilia, defects of liver function and kidney dysfunction) [10].

Recently, nanostructured lipid carriers (NLCs), has been introduced as a novel pharmaceutical dosage form derived from solid lipid nanocarriers (SLNs). They are also known as second generation of lipid nanoparticles [11, 12]. They have been extensively applied into oral, transdermal and intravenous drug delivery system [13] and are considered as a recent and efficient colloidal delivery system [14, 15]. NLCs have been introduced to overcome the limitation of SLNs i.e. drug loading capacity and drug leaking phenomena [16]. NLCs are composed of solid lipid matrix with certain percentage of liquid lipid. They are produced by controlled mixing of solid lipid with spatially incompatible liquid lipid which result in an imperfect matrix and results in high loading capacity [11, 17]. As liquid lipids have higher solubility for drugs, loading capacity of NLCs is higher than SLNs and also they provide controlled drug release. Additionally, due to lipidic nature and smaller size, NLCs have the capability to pass through GIT membrane in intact form and ultimately minimizing the contact of encapsulated drug with GIT membranes [18]. Also, NLCs have been suggested for specific applications such as cancer treatment, gene therapy, diagnosis and medical devices production [16, 19].

Due to convenient and safe administration of drug, transdermal drug delivery system (TDDS) has received greater attention, recently. Drug delivered through TDDS offer advantages like, avoid gastrointestinal degradation, bypass the hepatic first pass effect, low cost, non-invasiveness, continuous and constant drug concentration and reduces the frequency of administration particularly for shorter half-life drugs [20, 21]. NLCs are excellent candidates for the TDDS as they show minimal toxicity. Other important feature include skin penetration enhancement, protection against degradation, modified drug release, adhesiveness, provide skin hydration and lubrication. Also, NLCs showed prominently greater drug penetration through rat skin in vitro and higher area under the concentration–time curve in vivo [21, 22].

The present study aimed to fabricate ALP-loaded NLCs followed by their incorporation into HPMC based poloxamer-407 gel. The NLCs and NLCs gel were characterized physicochemical and were compared with conventional gel and ALP suspension. In vitro release and ex vivo permeation studies were executed for the optimized formulation and compared with ALP suspension, ALP conventional gel and ALP-loaded NLCs. Moreover, safety analysis and anti-gout study of the ALP-loaded NLCs gel was preformed was performed in Sprague–Dawley rat model.

### Chemicals and reagents

Stearic acid and potassium dihydrogen phosphate were obtained from BDH laboratory (Poole, England). Allopurinol, tween-20, poloxamer-407, hydroxy propyl methyl cellulose, oleic acid, eucalyptus oil, sodium chloride and sodium hydroxide were purchased from Sigma Aldrich (Steinheim, Germany). Disodium hydrogen phosphate was bought from Duksan (Ansan city, Kyunggi, Korea). Dialysis membrane tubes (12–14 kDa) was obtained from Membrane Filtration Products (Texas, USA). All other reagents used in this study were of pure analytical grade.

### Animals

Male Sprague–Dawley rats (weighing 270 ± 20 g) were purchased from Riphah institute of pharmaceutical sciences, Islamabad, Pakistan and were used in anti-gout and skin irritation study. They were placed in animal house with drinking water facility and standard animal food. Additionally, 24–25 °C temperature was maintained along with 50–60% relative humidity. The procedures used for performing animal studies were adopted from National Institutes of Health guide for the care and use of Laboratory animals (NIH Publications No. 8023, revised 1978), with the approval of Bioethical committee of Quaid-i-Azam University authorization approval number BEC-FBS-QAU2020-247. Moreover, all the animal studies executed in this research were in accordance with the ARRIVE guidelines.

### Preparation of ALP-loaded NLCs

Micro-emulsion method with some modification was used to fabricate ALP-loaded NLCs. Briefly, both the lipids (stearic acid and oleic acid) along with the drug (ALP) were heated up to 85 °C, using a hot plate (MAGIK MG-855), in order to obtain a uniform oily phase. Meanwhile, aqueous phase was obtained by dispersing surfactant (Tween-20) in preheated (85 °C) double distilled water. Aqueous phase containing the surfactant was then disseminated slowly in the oily phase with continuous stirring at 800 rpm for 60 min under a magnetic stirrer. The temperature of the system was maintained at 85 °C. The obtained pre-emulsion was then subjected to homogenization via high shear mixer (D-91126, Heidolph, Germany) at 8000 rpm for 12 min. The resulting O/W micro-emulsion was dispersed in chilled (4 °C) double distilled water in quantity of 1:9 (micro-emulsion: water) in order to obtained ALP- loaded NLCs dispersion [23, 24].

### Optimization of ALP-loaded NLCs

Optimization of ALP-loaded NLCs was carried out via design Expert version 12 (Box Bhenkhen model). The proportion of stearic acid (solid lipid), ALP and tween 20 were varied and its effect was assessed in terms of mean particle size, charge on particles and % EE [25].

## Characterization of ALP-loaded NLCs

### Particle Size, poly-dispersity and zeta Potential Analysis

Particle size, poly-dispersity index (PDI) and zeta potential of ALP-loaded NLCs dispersion were determined via zeta sizer ZS90 furnished with a He–Ne laser that operate at a wavelength of 635 nm. All the measurements were carried out at a fixed light incidence angle 90^0^ and 25 °C with software version 6.34 (Malvern Instruments, Worcestershire, UK). Before analysis, 10 μL of ALP-loaded NLCs was dispersed in 1 mL of de-ionized water followed by vortexing for 1 min [26, 27]. After that, the sample was introduced into the cuvette for analysis.

### Entrapment efficiency of ALP-loaded NLCs

Entrapment efficiency of ALP- loaded NLCs was determined using in-direct method (by quantifying the amount of free drug in the supernatant) [28]. One mL from the prepared ALP-loaded NLCs was centrifuged at 14,000 rpm for 90 min at 4 °C. The supernatant obtained was diluted appropriately in acetonitrile at ratio of 1:10 (0.5 mL of supernatant in 5 mL acetonitrile). The amount of free drug was then measured via UV–visible spectrophotometer (HALO DB-20.UV–VIS Double Beam Spectrophotometer) at a wavelength of 252 nm.

Following equation was used to calculate the percent EE [29].

% entrapment efficiency $$=\frac{\mathrm{Wt}-\mathrm{Wf}}{\mathrm{Wt}}$$ ×100.

Where Wt = Total quantity of drug added and Wf = Quantity of free drug in supernatant**.**

### Morphological analysis of ALP-loaded NLCs

TEM (Hitachi, Japan) was used for analyzing the morphology of ALP-loaded NLCs. A drop of sample was adsorbed on carbon coated copper grid. The film on the grid was negatively stained via addition of 2% of phospho-tungstic acid solution (w/w), immediately. An accelerated voltage of 100 kV was used to observe the grid [30, 31].

### Powder x-ray diffractometer (PXRD) analysis

Prior to solid state characterization, ALP-loaded NLCs were lyophilized via freeze-dryer (SP Scientific, Warminster, PA). The crystalline nature of lyophilized ALP-loaded NLCs was assessed via X-ray diffractometer. PXRD patterns of pure ALP, stearic acid and ALP-loaded NLCs were recorded with an X-ray diffractometer (BruckerAxs, Germany). The system was equipped with Cu-Kα radiation. Analysis was performed at 40 kV voltage using a 30 mA current. All the samples were scanned in a 2θ angle range between 10° and 80° at a scanning rate of 3°/min and a step size of 0.02° [32, 33].

### FTIR analysis

To characterize the molecular dynamic of formulation and its individual component, FTIR analysis was carried out. FTIR spectrophotometer (Eco Alpha II- Bruker, Billerica, MA, USA) was used to acquire the FTIR spectra of ALP, stearic acid, oleic acid, their physical mixture and ALP-loaded NLCs. The FTIR spectra’s for all the ingredients and formulation were obtained in a range of 500–4000 cm^−1^. Analysis was performed at room temperature in triplicate [30, 34].

### Fabrication of ALP-loaded NLCs gel

ALP-loaded NLCs gel was fabricated using Hydroxy-propyl methylcellulose (HPMC) and Poloxamer-407. Briefly, 2 g of Poloxamer-407 was dissolved in 5.5 mL of water and was kept in refrigerator for overnight in order to dissolve completely. HPMC (200 mg) was dissolved in 3.5 mL of hot water. Then, optimized ALP-loaded NLCs were added with continuous stirring. After that, eucalyptus oil was added as permeation enhancer to HPMC drug mixture. Afterward, Poloxamer-407 solution was added to it with continuous stirring. Finally, water was added to make the final volume 10 g [35].

## Characterization of ALP-loaded NLCs gel

### Homogeneity test

Homogeneity of ALP-loaded NLCs gel was performed via visual examination for any visible particle, bubbles and lumps. Gel consistency was confirmed via pressing gel between thumb and index finger and it was observed whether gel is homogeneous or not [36].

### Drug content

One gram of ALP-loaded NLCs gel was dissolved in 100 mL of acetonitrile. The prepared solution was then subjected to sonication and filtration. Afterward, sample was analyzed via UV spectrophotometer to determine drug content [36].

### Spreadability study

Spreadability study of ALP-loaded NLCs gel was performed via glass slide method. Briefly, two slides were taken and center of one glass slide was marked with a circle of 1 cm diameter. Gel (0.5 g) was placed with in the marked circle. Then, the second slide was kept over the first one. A weight of 500 g was placed over the upper slide for 5 min. Weight was removed after 5 min and increase in diameter was noted. Following formula was used to determine Spreadability index: $\mathrm{Si}=\mathrm{d}2\times\uppi /4$

Where Si= Spreadability index and d is the diameter [37].

### Measurement of pH

Determination of gel pH is of prime importance in respect to the application of formulation on skin. pH of the ALP-loaded NLCs gel was determined by dipping pH meter rod in the formulation [37].

### Effect of gel on environment pH

The effect of gel on pH of environment was checked by adding 1 g of gel in buffer pH 5.5 and pH was measured after 0.5, 1, 6 and 24 h [38].

### Measurement of bio-adhesive strength

Modified balance method was used for the evaluation of bio-adhesive strength of ALP-loaded NLCs gel. Rat having weight of 270 g was sacrificed and skin was removed. Hairs were shaved and the underlying loose tissues and fats were removed from the skin. Two pieces of skin (each 3 cm^2^) were obtained and were washed with PBS 7.4. Simultaneously, two glass vials (10 mL) were taken and were positioned such that one glass vial was attached to the reframed balance upside down, whereas the 2^nd^ glass vial was placed on an adjustable pan in upright position using double adhesive tape. One piece of the skin tissue was attached to the upside down glide slide where’s the other skin tissue was placed on the upright glass slide. Then, 0.5 g ALP-loaded NLCs gel was applied on the lower (upright glass slide) and it was adjusted, using adjustable pan, such that both the glass vials gently attached each other. Then, weights were placed in an ascending order on the other side of the balance, until the detachment of the two slides occur [39, 40]. The weight that was required to detach the two glass vials was noted as the bio-adhesive strength.

Following formula was used for calculation of bio-adhesive strength,

B.S = *WA.*

Where, B.S is bio-adhesive strength, W, is weight required (g) and A is area (cm^2^).

### Stability study of ALP-loaded NLCs

Stability study was conducted according to international conference of harmonization (ICH) guidelines Q1A (R2). The ALP-loaded NLCs were subjected to two different temperatures, 40 °C ± 2/ 75% RH ± 5% RH (accelerated stability testing, general class) and 25 °C ± 2/ 60% RH ± 5% RH (accelerated stability testing, substances to be stored in refrigerator) for 6 months. After storage at specific conditions, samples were analyzed for particle size, PDI, zeta potential and EE% at designated time intervals (0, 1, 3 and 6) months [41, 42].

### In vitro release studies

The prepared ALP-loaded NLCs were subjected to *in vitro* release study at pH 5.5 and 7.4. Dialysis bag method was used to perform *in vitro* release study. ALP-loaded NLCs gel containing ALP equivalent to 3 mg was used in this study and was compared with ALP suspension, ALP conventional gel, and ALP-loaded NLCs having equivalent amount of drug. Briefly, each formulation was poured into dialysis bag with both end fixed by thread and was placed in beakers filled with 50 mL pre-heated dissolution media. The beakers were then placed in a water bath maintained at 37 ± 1°C and horizontal shaking of 75 rpm. Two mL sample was collected at fixed time interval and same amount of fresh media was added accordingly. The collected samples were then observed spectrophotometrically at a wavelength of 252 nm and amount of released drug in each sample was calculated via comparing with concentration from standard curve [43].

### Skin irritation study

Skin irritation study was performed on rats to exhibit the safety of ALP-loaded NLCs gel after their transdermal application. Rats were divided into three groups and hairs were shaved from their dorsal side. Group I was treated with formalin 0.8% (Positive control), group II was treated with ALP-loaded NLCs gel and group III was treated with normal saline (Negative control). After the application of respective formulation rat skin was observed for erythema and edema for 24 h. Draize scoring method was used for the determination of primary dermal irritation index (PDII). After 24 h, rats were sacrificed via spinal dislocation and respective skin area was removed surgically and stored in 10% formalin. Then H & E slides were prepared from the stored skin area for histopathological examination [10, 44].

### Skin permeation study

The in vitro skin permeation study of ALP-loaded NLCs gel and ALP conventional gel was carried out via Franz diffusion cell apparatus (Premerger, USA) [45]. Rat skin was used for the permeation study. Rats were sacrificed; skin was shaved and then removed surgically. The skin after surgical removal was washed with PBS and stored at -20 °C. After 7 days of the skin isolation, the rat skin was taken out from the freezer, soaked in PBS for 30 min at 37 °C prior to use and then fixed between the donor and receptor compartment with dermal site facing toward receptor chamber. The capacity of receptor chamber was 5 mL with 0.77 cm^2^ area. The receptor chamber was filled with PBS 7.4 and the temperature was maintained at 37 ± 0.5 °C. Gel weighing 0.5 g was placed in the donor chamber and sample were collected at predetermined time (0.5, 1, 1.5, 2, 3, 4, 6, 12 and 24 h) and were replaced with same volume of fresh buffer. The samples were analyzed for the amount of drug permeated via UV spectrophotometer at a wavelength of 252 nm. Following equation were used to calculate the permeation parameters;

Flux (J) = $$\frac{Amount of drug permeated}{Time \times area of the membrane}$$ [46].

Kp = *J*/*C* [27].

ER = Kp of ALP-loaded NLCs gel / Kp of ALP conventional gel.

Where Kp: Permeability coefficient, J: Flux, C: Concentration of drug in donor chamber.

ER: enhancement ratio [47].

### Preparation of mono sodium urate (MSU) crystals

To prepare MSU crystals, 1 g of uric acid was dissolved in 200 mL of boiling water containing 8.12 mL of 1 normal NaOH. HCl was used to adjust the pH to 7.2 and the solution was then stored overnight at 4 °C. After overnight storage, the solution was subjected to heating (60 °C) in order to evaporate the solvent and obtain the crystals. The obtained crystals were sterilized in a tray dryer for 2 h at 180 °C and stored in sterile area till further use [48].

### In vivo anti-gout study

Male Sprague Dawley rats weighing 270 ± 20 g were divided into 3 groups having 6 rats in each group. Gout in rats was induced by the introduction of MSU (30 mg/mL) crystals via intra-synovial injection. Redness and swelling confirmed the development of gout. After 7 days of MSU injection treatment was started accordingly. Group II received ALP suspension via oral route at a dose of 10 mg/ kg. Group III received ALP-loaded NLCs gel via transdermal route at a dose of 5 mg/kg. Group I received no treatment. The diameter of knee joint was measured via Vernier caliper to evaluate inflammation. X-ray radiograph of knee joint were compared with the normal in order to assess level of deposition and degradation of MSU crystals [49].

## Results

### Fabrication and optimization of ALP-loaded NLCs

ALP-loaded NLCs were successfully prepared by micro-emulsion method The formulation was optimized via Design Expert by changing the proportion of solid lipid (stearic acid), amount of surfactant (tween-80) and drug (ALP) to assess their effects on particle size, zeta potential and % EE. The results for all three variables were significant with value of *P* < 0.05. The effects of changing variables on the properties of ALP-loaded NLCs are depicted in Fig. 1 and Table 1. F2 was selected as optimized formulation on the basis of smaller particle size (238.1 ± 3.1 nm), uniform distribution with PDI of 0.115, suitable zeta potential of -31.5 mV ± 1.1 mV and excellent %EE of 87.3% ± 1.16.

**Fig. 1:** Response surface 3D plots, Effect of surfactant, solid lipid and drug on particle size (A I, II, III); Zeta potential (B I, II, III); and entrapment efficiency (C I, II, III)

**Table 1:** Optimization chart of the allopurinol loaded nano lipid carrier (ALP-loaded NLCs)

		**Factor 1**	**Factor 2**	**Factor 3**	**Response 1**	**Response 2**	**Response 3**
**Standard deviation**	**Run**	**Stearic acid** **(mg)**	**Allopurinol** **(mg)**	**Tween-20** **(mg)**	**PS (nm)**	**ZP (mV)**	**EE (%)**
11	1	8	1	1.5	260.01 ± 2.3	-23.6 ± 0.8	74.1 ± 1.3
1	2	7	1	1	238.13 ± 3.1	-31.5 ± 1.10	87.3 ± 1.1
3	3	7	2	1	262.07 ± 4.3	-39.5 ± 1.14	75.1 ± 1.6
10	4	8	2	0.5	289.1 ± 2.9	-33.1 ± 0.87	61.2 ± 1.7
4	5	9	2	1	330.8 ± 3.6	-36.00 ± 1.4	55.7 ± 2.1
13	6	8	1.5	1	275.04 ± 3.2	-36.4 ± 0.93	68.1 ± 1.5
5	7	7	1.5	0.5	270.09 ± 3.3	-33.7 ± 1.21	70.3 ± 1.8
6	8	9	1.5	0.5	323.3 ± 4.3	-33.9 ± 1.10	50.5 ± 1.8
7	9	7	1.5	1.5	255.12 ± 1.9	-35.5 ± 0.96	78.3 ± 2.5
9	10	8	1	0.5	270.07 ± 3.7	-36.1 ± 1.30	66.1 ± 1.6
8	11	9	1.5	1.5	305.01 ± 4.3	-36.5 ± 1.23	57.0 ± 1.1
12	12	8	2	1.5	268.3 ± 3.9	-43.9 ± 0.76	64.0 ± 2.0
14	13	8	1.5	1	273.45 ± 4.1	-35.9 ± 1.42	67.5 ± 1.31
2	14	9	1	1	292.32 ± 3.8	-30.6 ± 0.31	63.6 ± 0.9

All the values here represent mean ± standard deviation

*PS* Particle Size, *EE* Entrapment efficiency, *ZP* Zeta Potential, *mg* Milligram, *nm* Nanometer, *mV* Millivo*lt*

### Particle size, PDI, zeta potential and entrapment efficiency

Dynamic light scattering analysis showed that the mean particle size of optimized ALP-loaded NLCs was 238.1 ± 5.3 nm, confirming that the formulation was of nano-size range. The PDI value of 0.169 confirmed that the size distribution of formulation was mono-dispersed (Fig. 2a). The zeta potential analysis showed that the optimized formulation had a negative charge of -31.5 ± 1.2 mV on its surface, signifying the stable nature of ALP-loaded NLCs (Fig. 2b). The %EE of the optimized ALP-loaded NLCs was 87.24%.

**Fig. 2:** Particle characterization. **A** Particle size and PDI analysis. **B** Zeta potential analysis. **C** TEM analysis

### Morphology of ALP-loaded NLCs

TEM analysis was performed in order to check the surface morphology of the ALP-loaded NLCs It was observed that the ALP-loaded NLCs particles has spherical shape and smooth surface morphology. The results also showed clear boundaries between the particles and particles were well segregated, indicating the stable nature of ALP-load NLCs. The results also showed that ALP-loaded NLCs had a mean particle size below 250 nm. TEM results were in accordance with the DLS analysis, demonstrating the formation of mono dispersed nano sized particle. (Fig. 2c).

### PXRD analysis

Polymorphic changes in drug and solid lipid were assessed via PXRD. X-ray diffractogram of ALP displayed certain diffraction peaks at 2θ equal to 11.98°, 14.76°, 17.301°, 24.33°, 25.68° and 28.11°, conforming the crystalline nature of ALP. These results were according to PXRD pattern of ALP reported in literature [5]. Likewise, stearic acid showed peaks at 2θ equal to 21.7° and 24.3°, demonstrating its crystalline nature as reported earlier in literature [50]. However, when incorporated and processed together in the ALP-loaded NLCs, these diffraction peaks were absent in the X-ray diffractogram of ALP-loaded NLCs. This study confirms the alteration of crystalline drug to amorphous form after encapsulation of ALP into the NLCs using nano formulation technique (Fig. 3).

**Fig. 3:** PXRD analysis of pure Allopurinol (ALP), Stearic acid and ALP-loaded NLCs

### FTIR analysis

Intermolecular interactions between ALP and formulation ingredients were assessed via FTIR analysis. Figure 4 depicts the FTIR spectra of ALP, stearic acid, oleic acid, physical mixture and ALP-loaded NLCs. The FTIR spectrum of ALP showed principle peaks at, 2986 cm^−1^ demonstrating CH stretching of the pyrimidine ring, 1763 cm^−1^ representing C = O stretching of the keto form of the 4 hydroxy tautomer, 1226 cm^−1^ and 778 cm^−1^ signifying CH stretching in plane deformation, 1580 cm^−1^ indicating ring vibration. Oleic acid showed corresponding peaks at 2922 cm^−1^ indicating asymmetric CH_2_ stretching, 2853 cm^−1^ indicating symmetric CH_2_ stretching, 1708 cm^−1^ indicating C = O stretching, 1412 cm^−1^ indicating OH stretching in plane, 1285 cm^−1^ indicating C-O stretching, 935 cm^−1^ indicating OH stretching out of plane. The spectrum of stearic acid showed distinctive peaks at 2955 cm^−1^, 2847 cm^−1^, 1697 cm^−1^, 1294 cm^−1^, 721 cm^−1^ demonstrating OH, CH and C = O stretching.. FTIR spectra of ALP-loaded NLCs demonstrated all the representative peaks of ingredients, assuring the absence of any chemical interaction between the lipids and drug.

**Fig. 4:** FTIR analysis of pure Allopurinol (ALP), Stearic acid, Oleic acid, Physical mixture and ALP-loaded NLCs

### Preparation and characterization of ALP-loaded NLCs gel

The ALP-loaded NLCs gel was prepared by using HPMC and Poloxamer-407. The gel was milky white in appearance and was free of any gritty particle and lumps indicating the homogeneity of the gel. The pH of the gel was 6.13 ± 0.09. The ALP-loaded NLCs gel showed drug content of 97.3% ± 1.5% and high spreadability of 391 ± 8.2 mm^2^. Moreover, the ability of gel to bind to a biological membrane surface is very important parameter was thus investigated for the prepared gel. The bio-adhesive strength of prepared HPMC based poloxamer-407 gel was found to be 9806.65 Dyne/cm^2^. This Bioadhesive strength may help the gel to remain on biological membrane surface after its application and extend its drug release over a sufficient period of time.

### Skin irritation study

The skin irritation was evaluated on the bases of Draize scoring. PDII score was used for indicating erythema and edema. The results of skin irritation study are shown in Fig. 5 and Table 2. In formalin treated group, clear erythema and edema can be seen as marked by circle and arrows in Fig. 5a I. The PDII (calculated from PDI) for this group was 4.33, indicating moderate irritation. ALP-loaded NLCS and normal saline treated groups showed no edema and erythema (Fig. 5a II & III). These groups had a PDII of 0.33 and 0, respectively and indicated negligible and no irritation, correspondingly (Table 2). The skin irritation study results were further supported by the histopathology analysis. The histopathological results of skin irritation study indicated skin tissue damage in case of 0.8% formalin treated group (indicated by arrows in Fig. 5b I). Major infiltration and inflammation can be seen in 0.8% formalin treated group. However, no such skin tissue damage or inflammation was seen in the ALP-loaded NLCs gel and normal saline treated group (Fig. 5b II & III).

**Fig. 5:** Skin irritation study in Sprague–Dawley rats, after dermal application (**A**), and Histopathological analysis (**B**) of 0.8% Formalin treated group, ALP-loaded NLCs gel treated group and untreated control group. Bar length shows 50 µm. Arrows and circles in 5A I represents erythema and edema, while in 5A II and III arrows represents absence of erythema and edema. Arrows in 5B I, shows dermal damage

**Table 2:** Skin irritation study using Draize scoring of formalin treated and gel treated rats as compared with untreated rats

	**Time (hrs)**	**Untreated rat** **(Control)**	**Formalin** **Treated rats**	**ALP-loaded NLCs** **Treated rats**
**Erythema**	1	0	3	1
	12	0	3	0
	24	0	2	0
**Edema**	1	0	1	0
	12	0	2	0
	24	0	2	0
**PDI**	1	0	4	1
	12	0	5	0
	24	0	4	0
**PDII**		0	4.33 (Moderate)	0.33 (Non-significant)

*PDI Primary dermal irritation, PDII Primary dermal irritation index*

## Stability study of ALP-loaded NLCs

The stability study of ALP-loaded NLCs was conducted for 6 months at two different temperatures to evaluate the outcome of storage condition on physiochemical properties of the formulation. The results of stability study showed no significant changes in particle size, PDI, zeta potential and EE% at both the temperature (Table 3). At 25 °C the particle size was changed from 238.1 nm to 247.7 nm, PDI from 0.115 to 0.121, zeta potential from -31.5 to t0 -30.2 and %EE from 87.3% to 84% within a period of 6 months. All these changes were non-significant. Also at 40 °C, non-significant changes in particle size from 238.1 to 250.2, PDI from 0.115 to 0.129, zeta potential from -31.5 to -29.3 and %EE from 87.3 to 83.17 were observed.

**Table 3:** Stability study of the optimized ALP-loaded NLCs as per the International conference of harmonization (ICH guidelines)

**Storage temperature**	**25 °C ± 2**^a^				**40 °C ± 2**^b^			
**Relative humidity**	**60% RH ± 5% RH**				**75% RH ± 5% RH**			
**Time (months)**	**0**	**1**	**3**	**6**	**0**	**1**	**3**	**6**
**Particle size (nm)**	238.1 ± 5.3	240.3 ± 5.4	243.9 ± 5.8	247.7 ± 5.8	238.1 ± 5.3	241.5 ± 5.5	245.6 ± 5.2	250.2 ± 5.8
**Zeta potential (mV)**	-31.5 ± 1.2	-31.0 ± 2.2	-30.8 ± 1.8	-30.2 ± 1.8	-31.5 ± 1.2	-30.6 ± 2.0	-30.1 ± 1.5	-29.3 ± 1.8
**PDI**	0.115 ± 0.02	0.118 ± 0.02	0.119 ± 0.03	0.121 ± 0.05	0.115 ± 0.02	0.117 ± 0.01	0.124 ± 0.02	0.129 ± 0.04
**Entrapment efficiency** **(%)**	87.3 ± 1.3	85.9 ± 1.4	85.19 ± 1.5	84.11 ± 1.5	87.3 ± 1.3	85.16 ± 1.4	84.54 ± 1.7	83.17 ± 1.5

All the values here represent mean ± standard deviation; *n* = 3

*PDI* Polydispersity Index, *nm* Nanometer, *mV* Millivolt

^a^Represents the accelerated storage condition for the substance to be stored in refrigerator

^b^Represents the accelerated storage condition for general class

### In vitro drug release and release kinetic models

In vitro release characteristics of ALP from ALP suspension, ALP conventional gel, ALP-loaded NLCs and ALP-loaded NLCS gel were checked at two different pH (pH 5.5 and 7.4) environments in the relevant media. At both the pH values, rapid release was observed in case of ALP suspension and ALP conventional gel as compared to ALP-loaded NLCs and ALP-loaded NLCs gel. At pH 7.4 (Fig. 6A), ALP suspension showed a release of 89% in the first 2 h. ALP conventional gel showed 42.99% drug release in first 2 h followed by 73.98% release in 6 h. Complete drug released was observed in 12 h from ALP conventional gel. While ALP-loaded NLCs and ALP-loaded NLCs gel showed a 17.12% and 11.44% release in initial 2 h followed by 37.58 and 22.54% release in 6 h. At 24 h period a release of 68.68% and 53.85% was observed from ALP-loaded NLCs and ALP-loaded NLCs gel, respectively. These results suggested that both ALP-loaded NLCs and ALP-loaded NLCs gel sustained the release of the drug. However, more sustained release behavior was observed in case of ALP-loaded NLCs gel as compared to ALP-loaded NLCs. At pH 5.5, ALP suspension showed a release of 76% in initial 2 h and complete drug was released in 6 h. ALP conventional gel showed 27.06% and 52.07% release in 2 and 6 h, respectively. A release of 89.12% was observed from ALP-loaded gel in 24 h. ALP-loaded NLCs and ALP-loaded NLCs gel showed 3.84% and 2.4% release in 2 h and 6.28% and 4.49% release in 6 h, respectively. At 24 h period, a release of 10.17% and 6.08% was observed from ALP-loaded NLCs and ALP-loaded NLCs gel, respectively (Fig. 6B).

**Fig. 6:** Cumulative in vitro release study of the ALP suspension, ALP conventional gel, ALP-loaded NLCs and ALP-loaded NLCs gel at pH 7.4 (**A**) and pH 5.5 (**B**). Data shows mean ± S.D. (*n* = 3)

Different kinetic models (Higuchi, Korsmeyerpeppas, 1st order, Zero order, Hixon Crowell) were applied to evaluate the best fit model. The results suggested that release from both the ALP-loaded NLCs and ALP-loaded NLCs gel followed korsmeyerpeppas (High R^2^ value) model (Table 4).

**Table 4:** Kinetics of drug release from ALP conventional gel, ALP-loaded NLCs and ALP-loaded NLCs gel

**R**^**2**^** value**	**Kinetic Model applied**				
	**Higuchi**	**Korsmeyer- peppas**	**Ist order**	**Zero order**	**Hixon-Crowell**
**ALP-loaded NLCs**	0.4937	0.9795	0.1285	-1.2676	-0.0936
**ALP-loaded NLCs gel**	0.8324	0.9805	0.3053	-2018	0.1537
**R**^**2**^** value for ALP conventional gel**	0.8145	0.9821	0.3211	-2103	0.1465

## Ex vivo permeation study

Ex vivo permeation study was conducted to evaluate the potential of ALP-loaded NLCs to cross the major skin barrier (stratum corneum) for transdermal drug delivery. The cumulative amount of ALP permeated/ area from ALP-loaded NLCs gel and ALP conventional gel was plotted against time (Fig. 7). ALP-loaded NLCs gel showed permeation of 269.4 µg /cm^2^ in initial 2 h and 463.19 µg /cm^2^ in 6 h. Maximum permeation of 863 µg /cm^2^ was observed in case of ALP-loaded NLCs gel. ALP conventional gel showed permeation of 10.98 µg /cm^2^ and 20.94 µg /cm^2^ in initial 2 h and 6 h, respectively. At a period of 24 h, permeation of 31 µg /cm^2^ was observed from ALP conventional gel. These results confirmed the excellent permeation of ALP-loaded NLCs as compared to ALP. Permeation parameters (steady state flux, permeability coefficient and enhancement ratio) were calculated from ex vivo permeation data (Table 5). The ALP-loaded NLCs showed 28 times enhanced permeation as compared to the free ALP as revealed by the enhancement ratio.

**Fig. 7:** Ex vivo permeation study of the ALP conventional gel, and ALP-loaded NLCs gel. Data shows mean ± S.D. (*n* = 5)

**Table 5:** *Ex- vivo* skin permeation parameters of ALP-loaded NLCs gel as compared to conventional gel

	**ALP-loaded NLCs gel**	**ALP conventional gel**
Flux (µg/cm^2^/hr)	46.699 ± 1.76	1.677 ± 0.10
PC	0.0467 ± 0.005	0.00168 ± 0.001
ER	27.84 ± 0.78	––

### In vivo anti-gout study

The in vivo anti-gout study was evaluated in term of inflammation (by measuring knee diameter) and change in the interspace in knee joints (via X-ray analysis). Treatment was started at day ‘7’ after the induction of gout by MSU crystal, confirmed by swollen and inflamed joints. A significant reduction in knee diameter was observed in ALP-loaded NLCs gel treated group as compared to untreated and ALP suspension treated group Fig. 8 and Table 6. The untreated group showed a marked increase in knee diameter till the completion of the study (from 4.12 ± 0.20 mm to 8.53 ± 0.58 mm). After initiation of treatment, the knee diameter was reduced to normal in ALP-loaded NLCs gel treated group (from 4.39 ± 0.38 mm to 4.46 ± 0.37 mm) at a dose lower than that of the ALP suspension, which demonstrate change in knee diameters (from 4.09 ± 0.324 mm to 4.63 ± 0.27 mm). X-ray analysis was carried out to further confirm the results of the study, as reported in Fig. 8 (A, B, C). It can be seen that the narrowing of joint spaces occurred in the untreated rats group after induction of the gout (Fig. 8 A). However, when treated with the ALP-loaded NLCs gel, the broadening of joint spaces were observed as reported in Fig. 8 B, indicating the significant reduction in inflammation in ALP-loaded NLCs gel treated group as compared to un-treated group. Similarly, despite the enhanced quantity of drug used in ALP suspension, the joint spaces were not fully broadened in ALP suspension group and the narrow joint space may be seen in Fig. 8 C. This study exhibited that ALP-loaded NLCs gel showed a significant reduction in inflammation at a lower dose as compared to ALP-suspension. These results demonstrated that loading of ALP into NLCs had increased its efficacy.

**Fig. 8:** X-ray analysis of in vivo anti-gout study, (**A**) Gout induced un-treated group; (**B**) ALP-loaded NLCs gel treated group; (**C**) ALP suspension treated group. Arrows in Fig A I, II and III represents diminished intra-articular space and induction of gout. Arrows in Fig B and C (I, II and III) signifies increase in intra-articular space after successful treatment

**Table 6:** Anti-gout study (knee diameter) of the Sprague–Dawley rats after their treatment with ALP-loaded NLCs gel and its comparison with ALP suspension and untreated rats groups.

**Treatment group**	**Day (s)**				
	**0**	**7**	**15**	**30**	**45**
	**Knee diameter (mm)**				
**Gout induced untreated**					
GR1	4.11	8.42	8.46	8.48	8.49
GR2	3.92	7.90	7.91	7.93	7.92
GR3	3.84	7.74	7.77	7.79	7.80
GR4	4.45	8.75	8.76	8.78	8.77
GR5	4.30	8.61	8.63	8.66	8.64
GR6	4.12	9.53	9.52	9.55	9.56
**ALP suspension**					
SR1	3.83	7.67	6.31	5.43	4.39
SR2	4.22	8.23	6.94	6.01	4.89
SR3	4.43	8.54	7.07	6.13	4.97
SR4	4.56	8.47	7.19	6.26	4.85
SR5	3.70	7.64	6.08	5.40	4.24
SR6	3.85	7.79	6.21	5.33	4.48
**ALP-loaded NLCs gel**					
NGR1	3.78	7.94	6.21	5.07	3.84
NGR2	4.07	7.99	6.18	5.11	4.12
NGR3	4.63	8.47	6.72	5.79	4.67
NGR4	4.34	8.35	6.81	5.76	4.48
NGR5	4.71	7.89	6.57	5.69	4.80
NGR6	4.86	8.31	7.04	5.48	4.89

## Discussion

Herein, ALP-loaded NLCs were fabricated via micro emulsion method. This method was selected among various available methods for the preparation of NLCs, due to its simplicity, ease of production, less energy input required and owing to its easy process using common laboratory equipment’s. Stable NLCs with uniform particle size and mono-dispersed nature can be prepared via this method [51]. This technique has been successfully used for the preparation of aceclofenac NLCs with high entrapment and better stability [52]. Moreover, mefenamic acid loaded NLCs had also been prepared via this method successfully [53]. Apart from method of preparation, the formulation ingredient also affects the properties of NLCs. Stearic acid was selected as solid lipid due to its natural origin and high melting point which maintain the integrity of the NLCs formulation for longer time in harsh condition and provide stability to the NLCs [54]. Also, stearic acid has lighter and small fatty acid chain which results in NLCs with smaller particles size. Another important parameter for selecting stearic acid as solid lipid is its HLB value. Stearic acid has HLB value of [15] which is near to the HLB value of tween-20 (16.7) and will results in the production of stable NLCs formulation. Miscibility of the liquid and solid lipid is an important consideration [55, 56]. Oleic acid was selected as liquid lipid due to its excellent miscibility with stearic acid which ultimately results in the manufacturing of stable dispersion with uniform particle size. Also, various studies had reported high EE and smaller particle size with this combination [57, 58]. Tween-20 was selected as surfactant due to its non-ionic nature. Also, it improves the water solubility of insoluble moieties owing to its hydrophilic nature and its minimal toxicity to the biological membranes [59]. Tween-20 has HLB value of (16.7) which is suitable for o/w emulsion (most commonly used range is 8–18). ALP-loaded NLCs were optimized by using design expert version 12, Box Bhenken model by changing the concentration of solid lipid, ALP and tween 20. The effect of these variations was observed in term of particle size, entrapment efficiency (%EE) and zeta potential (Table 1). Figure 1A (I, II, III) demonstrated reduction in particle size as the concentration of solid lipid was decreased and that of liquid lipid and surfactant was increased. This reduction in particle size may be because of reduced viscosity and interfacial tension which results in smaller particle size with smooth surface [60, 61]. Increased drug concentration resulted in enlarged particle size owing to the augmented viscosity of the melted lipid. It has been reported earlier that a high viscosity has the tendency to form non uniform dispersion, leading to formation of larger particle size [57].

The stability of nanoparticle could be attributed to the surface charge over the nanoparticles. The value of zeta potential greater than ± 25 indicates the stable nature of the nanoparticles. Increase in zeta potential value of ALP-loaded NLCs was observed with increasing drug concentration, which may be attributed to negative charge on the surface of ALP [62]. Also, increase in zeta potential was observed by decreasing the solid lipid concentration and increasing the surfactant concentration. This increment in zeta potential value may be credited to reduction in particle size which increases the charge density on the surface of nanoparticle Fig. 1B (I, II, III) [61, 62]. Figure 1C (I, II, III) showed the effect of drug, lipid and surfactant concentration on the %EE. An enhancement in %EE was observed with reduction of solid lipid and increment in surfactant concentration. The reduction in solid lipid may ultimately results in enhancement of liquid lipid, which increases the solubility of drug in NLCs matrix and also results in crystal order disturbance leading to many imperfections in NLCs matrix and hence increased the %EE [57]. Increased %EE with high surfactant concentration may be because of the reduced interfacial tension between lipid and drug [63]. On the other hand, decreasing trend in %EE was observed with higher drug concentration due to the fact the quantity of lipid being not enough to accommodate higher drug concentration [64].

Morphological analysis via TEM validated the particles of NLCs in nano-metric size with globular shape, clear boundaries and no sign of aggregation, suggesting the stable and mono-dispersed nature of the particles [65]. The formulation properties were also influenced by the polymorphic form of the drug and lipid matrix. PXRD analysis was performed to check the polymorphic form of the components and the results showed that the ALP and stearic acid had characteristic crystalline peaks owing to their crystalline nature. Although, such crystalline peaks were absent in ALP-loaded NLCs demonstrating the transformation of crystalline ALP into amorphous one., owing to its entrapment in the NLCs matrix [66].

The FTIR spectrum of ALP demonstrated CH stretching of the pyrimidine ring, C = O stretching of the keto form of the 4 hydroxy tautomer, CH stretching in plane deformation and ring vibration [5]. Oleic acid showed asymmetric CH_2_ stretching, symmetric CH_2_ stretching, C = O stretching, OH stretching in plane, indicating C-O stretching and OH stretching out of plane[67]. The spectrum of stearic acid showed OH, CH and C = O stretching [68]. The FTIR spectrum of ALP-loaded NLCs validated the existence of all the listed functional groups, demonstrating no chemical interaction between the components of the formulation.

Bio-adhesive gels have excellent accessibility, ease self-placement of dosage and also provide easy application, localization and removal. HPMC was selected due to its non-toxic nature, swelling properties, control the release of the drug and are preferred for topical route due to its non-irritant nature. Poloxamer-407 is a non-toxic triblock co-polymer. Its aqueous solution is clear liquid at room temperature at refrigerator temperature and undergoes sol–gel transition and form gel when warmed to room temperature. Slow release characteristics are achieved from drug containing solutions due to this reverse thermal gelation. Addition of HPMC into Poloxamer-407 will not only modulates rheological and mechanical properties but also its gelation temperature [35, 69]. To increase the permeation of drug across the epithelium, the use of penetration enhancer is a logical approach. So eucalyptus oil was used as permeation enhancer [70]. The prepared ALP-loaded NLCs gel was milky white in color due to the addition of formulation which was milky white in color. The gel was homogenously dispersed without any gritty particles and the drug content was 97.3% ± 1.5% indicating uniform dispersion of the drug [71]. The spreadability of ALP-loaded NLCs gel was suitable enough to spread the gel on the site of application [72]. The pH of ALP-loaded NLCs gel was 6.13 ± 0.09 as the reported skin pH value ranges from 6–7.5 indicating that ALP-loaded NLCs gel in this pH range are appropriate for skin application [73].

Draize scoring method was used for the determination of skin irritation (Table 3). The PDII was calculated on the basis of erythema and edema presence. A score of zero represents no edema and erythema, 1 represents very slight, 2 slight, 3 moderate and 4 represent severe erythema and edema. PDI value was calculated by the average erythema and edema at that specific interval. PDII was calculated from PDI value (By dividing PDI score at all interval/ number of intervals). PDII value of 0–0.4 show negligible irritation, > 0.5–1.9 show slight irritation, 2- 4.9 show mild and > 5 show severe irritation. The ALP-loaded NLCs gel showed a negligible edema and erythema and no skin flare were observed, while 0.8% formalin treated group showed marked edema and erythema. The findings of the histopathological examination indicated damage of epidermal tissues in case of formalin treated group while no such damage was observed in case of ALP-loaded NLCs gel [36]. The findings of skin irritation study confirmed that ALP-loaded NLCs gel was appropriate for dermal application and exhibited no sign of skin irritation.

ALP-loaded NLCs and ALP-loaded NLCs gel were evaluated for release behavior at different pH imitating skin and plasma environment. The release of ALP in case of suspension and conventional gel was higher at pH 7.4 as compared to pH 5.5, the reason behind this lower release at pH 5.5 is lower solubility of ALP at acidic pH [74]. Drug release from the ALP-loaded NLCs and ALP-loaded NLCS gel was minimal at skin PH, which is attributed protection provided by surfactant [75]. The ALP-loaded NLCS and ALP-loaded NLCS gel showed sustained release as compared to ALP conventional gel and ALP suspension**.** However, the ALP-loaded NLCs gel showed a more sustained release as compared to ALP-loaded NLCs. This sustained release of ALP from NLCs may be attributed to protection inside the core of lipid carriers [76]. The polymer in ALP-loaded gel acts as a competent reservoir to the formation of condensed gel matrix structure. As a result of entrapment of ALP in gel matrix, it has to experience an additional barrier, resulting in its sustained release. Through this type of release behavior high concentration gradient is achieved requisite for effective transdermal drug delivery [77]. The ex vivo permeation study demonstrated higher permeation of the drug across the rat skin for the ALP-loaded NLCs gel as compared to the ALP conventional gel. The permeation enhancer used, enhances drug permeation through skin by interacting with the lipid domain of stratum conium and creating channel for the drug to permeate. The permeation parameter (flux, permeability coefficient and enhancement ratio) were calculated from the permeation graph. The enhancement ratio was 27.84 time for ALP-loaded NLCs gel as compared to ALP conventional gel [78].

The anti-gout activity of ALP-loaded NLCs gel was significantly enhanced as compared to ALP suspension, despite using more drug concentration in suspension. There was a marked reduction in knee diameter in both ALP suspension and ALP-loaded NLCS gel treated group, however, the results of ALP-loaded NLCS gel were significant being at the lower drug concentration. The x-ray results also confirmed the reduction in inflammation characterized by broadening of intra-articular spaces. The results also showed the supremacy of ALP-loaded NLCs gel because the ALP-loaded NLCs gel produced better results in a lesser dose as compared to ALP suspension given orally. This higher efficacy may be attributed to the NLCs which make the drug solubilize and make the drug available at the sight of action. Another reason might be the sustained release of the drug from ALP-loaded NLCs gel which enhanced the efficacy of ALP. Also, the utilization of non-ionic surfactant results in enhanced permeation of the drug by working as a permeation enhancer and improved the therapeutic efficacy of ALP. The presence of lipids and surfactant results in a better interaction of the NLCs formulation with biological membrane and ensure its better availability at the site of action in comparison to the free drug which is water insoluble. The permeation enhancer used also enhances the drug permeation through the skin by interacting with the lipid domain of stratum conium and creating channel for the drug to permeate. There by increasing the availability of drug at sight of action and hence therapeutic efficacy [49].

## Conclusions

In present study, ALP-loaded NLCs were prepared with optimal particle size, PDI and zeta potential. The formulation was successfully optimized via design expert and characterized via TEM, XRD and FTIR. The prepared NLCs were then successfully loaded into HPMC Poloxamer-407 based gel and characterized successfully. The in vitro release studies confirm minimal release of drug on skin surface, whereas the ex vivo permeation study confirmed better permeation in case of ALP-loaded NLCs gel. Similarly, In vivo skin irritation study showed minimal irritation in case of ALP-loaded NLCs gel. The enhancement ratio for formulation gel was 28 times greater than the conventional gel. The ALP-loaded NLCs gel showed excellent anti-gout activity as compared to ALP suspension at a lower dose. Overall, this study showed the potential of ALP loaded NLCs for transdermal application with sustained release, minimal side effect and excellent anti-gout activity.

## Declarations

### Availability of data and materials

All data generated or analysed during this study are included in this published article.
